This article has been retracted.

# Detection of Abnormal Hemoglobin Variants by HPLC Method: Common Problems with Suggested Solutions

**DOI:** 10.1155/2014/257805

**Published:** 2014-10-12

**Authors:** Leela Pant, Dipti Kalita, Sompal Singh, Madhur Kudesia, Sumanlata Mendiratta, Meenakshi Mittal, Alka Mathur

**Affiliations:** ^1^Department of Pathology, Hindu Rao Hospital, Delhi 110007, India; ^2^Thalassemia Control cell, Hindu Rao Hospital, Delhi, India; ^3^Department of Pediatrics, Hindu Rao Hospital, Delhi, India

## Abstract

Thalassemia and thalassemic hemoglobinopathies pose serious health problem leading to severe morbidity and mortality in Indian population. Plethora of hemoglobin variants is prevalent in multiethnic Indian population. The aim of the present study was to analyze laboratory aspects, namely, hematological profile and HPLC findings of the hemoglobin variants detected, and to discuss problems that we faced in diagnosis in a routine clinical laboratory. We screened a total of 4800 cases in a hospital based population of North India in a 2-years period of by automated HPLC method using the Variant Hemoglobin Testing System (Variant II Beta Thalassemia Short Program, Bio-Rad Laboratories) under the experimental conditions specified by the manufacturer. Whole blood in EDTA was used and red cell indices were determined using automated hematology analyzer. We detected 290 cases with abnormal variants in which beta thalassemia was the most common followed by hemoglobin E. Here, we discuss the laboratory aspects of various hemoglobin disorders and diagnostic difficulties in cases like borderline HbA2 values, presence of silent mutation, alpha thalassemia gene, and few rare variants which at times require correlation with genetic study. Special attention was given to HbA2 level even in presence of a structural variant to rule out coinheritance of beta thalassemia gene.

## 1. Introduction

Thalassemia is an autosomal recessive inherited group of disorders of hemoglobin synthesis characterized by the absence or reduction of one or more of the globin chains of hemoglobin. The structural variants result from substitution of one or more amino acids in the globin chains of the hemoglobin molecule [1]. Plethora of hemoglobin variants is prevalent in India owing to ethnic diversity of its population with minimal to major clinical significance. Being recessively inherited from the parents, the thalassemia and thalassemic hemoglobinopathies pose serious health problem leading to severe morbidity and mortality in Indian population.

Detection of asymptomatic carriers by reliable laboratory methods is the cornerstone of prevention of this serious health problem. Cation exchange high performance liquid chromatography (CE-HPLC) has become the preferred technique suitable in Indian scenario, as it can detect most of the clinically significant variants. The simplicity of the automated system with internal sample preparation, superior resolution, rapid assay time, and accurate quantification of hemoglobin fractions makes this an ideal methodology for the routine clinical laboratory [2, 3].

With increasing global awareness and mass screening programs undertaken at various levels by health care system, the responsibility for laboratory personnel has greatly enhanced in detection and prevention of this problem. Awareness about the diagnostic problems as well as their solutions is very important so that one does not miss a single case.

Many studies have been published from India on thalassemia and thalassemic hemoglobinopathies mostly putting emphasis on epidemiology and screening [4–6].

Very few studies are available on the approach of diagnosis and problems in routine diagnosis, especially in laboratories with limited resources.

The aim of the present study was to analyze laboratory aspects, namely, hematological profile and HPLC findings of the hemoglobin variants detected, and to discuss problems that we faced in diagnosis in a routine clinical laboratory.

## 2. Material and Methods

This was a prospective study carried out in the Department of Pathology and Thalassemia Control Cell, Hindu Rao Hospital, Delhi, for 2 years' period. A total of 4800 cases were screened for presence of thalassemia or any structural variant. These included all cases of microcytic hypochromic anaemia (MCV < 80 fl, MCH < 27 pg, and RBC count > 5 million/*μ*l) not responding to conventional treatment, clinically suspected cases of hemoglobinopathy, antenatal, and other cases coming to the department for thalassemia screening. A 5 mL intravenous blood sample was collected in EDTA anticoagulant. Red cell indices were measured on an automated haematology analyzer (Sysmex KX 21).

HbA2, HbF, and other haemoglobin variants were studied by HPLC method used for chromatographic separation of human hemoglobin [7–9].

We used the Variant Hemoglobin Testing System (Variant II Beta Thalassemia Short Program, Bio-Rad Laboratories Inc., Hercules, CA, USA) under the experimental conditions specified by the manufacturer [10].

### 2.1. Principle

The Variant II Beta Thalassemia Short Program utilizes principles of ion-exchange high-performance liquid chromatography (HPLC). The samples are automatically mixed and diluted on the Variant II Sampling Station (VSS) and injected to the analytical cartridge. The Variant II Chromatographic Station (VCS) dual pumps deliver a programmed buffer gradient of increasing ionic strength to the cartridge, where HbA2/F are separated based on their ionic interaction with the cartridge material. The separated HbA2/F then pass through the flow cell of the filter photometer where the changes in absorbance at 415 nm are measured. An additional filter at 690 nm corrects the background absorbance. The Variant II CDM (CDM) Software performs reduction of raw data collected from each analysis. To aid in the interpretation of results, windows have been established for the most frequently occurring hemoglobins based on the characteristic retention time. For each sample a sample report and a chromatogram are generated by CDM showing all hemoglobin fractions eluted, their retention times, the area of the peaks, and values of the fractions.

### 2.2. Reagents

1. Elution buffers (1,2): sodium phosphate buffer.
2. Whole blood primer: lyophilized human red blood cell hemolysate with gentamicin, tobramycin, and EDTA as preservative.
3. HbA2/F calibrator/diluent set: lyophilized human red blood cell hemolysate with gentamicin, tobramycin, and EDTA as preservative analytical cartridge. Diluent contains deionized water.
4. Wash/diluent solution: deionized water.
5. Control: normal (HbF 1-2%, HbA2 1.8–3.2%) and abnormal (HbF 5–10%, HbA2 4–6%) controls.

### 2.3. Sample Collection and Preparation

Five milliliters (5 mL) of whole blood was collected in a vacuum collection tube containing EDTA which can be stored at 2–8 degrees C for maximum 7 days if processing is delayed. No preparation was required unless the sample was in a tube other than the recommended tube or there was less than 500 *μ*L of sample in the tube. In such case, sample was manually prediluted. Predilution was carried out by mixing 1.0 mL wash/diluents with 5 *μ*L of whole blood sample.

HbA2/F calibrators and normal and abnormal controls were analyzed at the beginning of each run.

### 2.4. Interpretation of Reports

Reports and chromatograms generated were studied and interpreted by observing HbA2 and F concentration for beta thalassemia and retention time and area percentage of other peaks and windows for structural variants. Each chromatogram shows peaks of Hb A0, A2, and Hb F along with C window, D window, S window, and two minor peaks, P2 and P3. Several hemoglobin variants elute same window; they were provisionally diagnosed by retention time and area percentage keeping in mind the ethnicity of the patients.

Other relevant tests were done, for example, sickling test as supporting evidence of Hb S. Family study was carried out whenever possible and correlation with findings of Hb electrophoresis result was done in few cases.

## 3. Results and Discussion

### 3.1. Results

Among 4800 cases screened, 290 (6.04%) cases were detected with abnormal hemoglobin in this study. Presumptive identification of hemoglobin variants was made primarily by retention time (RT) windows and area percent; however geographical factor, ethnicity, and clinical presentation were also taken into consideration. Distribution of hemoglobin variants identified is shown in Table 1. Their relevant RBC parameters and HPLC findings are given in Table 2. Chromatograms of some important variants are shown in figures (Figures 1, 2, 3, 4, 5, and 6).

Genotypes of some structural variants are shown in Table 3.

As expected, beta thalassemia trait (BTT) was the most common hemoglobin variant (74.48%) detected in our study with elevated HbA2 level (>3.5%) and RT 3.63–3.69 min. Majority were asymptomatic and detected during carrier screening and family studies.

Nine cases of beta thalassemia were detected which were classified as either major or intermedia depending upon clinical severity. HbF was raised (20.7–97.1%), with variable HbA2 (2.4–5.7%). Cases of thalassemia major presented within 1st year of life. Parental study was done to find out carrier status and to confirm the diagnosis.

Three cases showed raised HbF (13.7–19.7%), normal HbA2 values (2.2-2.3%), and normal Hb level, raised RBC count, and reduced MCV and MCH levels. Parental study was done with a provisional diagnosis of delta beta thalassemia trait and DNA study was advised.

Hemoglobin E (HbE) was found to be the most common structural variant with raised peak in A2 window (RT 3.76–3.78 min). A total of 28 cases of Hb E trait were detected with peak area ranging from 18.5 to 39% and mild elevation of HbF level. Two cases of homozygous Hb E were detected showing 77–83% HbE and 2–5% HbF. Hb level was mildly reduced with raised RBC counts and reduced MCV and MCH values. Parental study was carried out for confirmation.

Two cases of double heterozygous of HbE and beta thalassemia trait were found showing peak in HbA2 window (53.5–69.7%) and raised HbF level (5–14.5%). Again, parental and family study was carried out for confirmation.

Nineteen cases showed peak in the D window (RT 4.13–4.15 min), indicating presence of structural variant hemoglobin D (Hb D) Punjab. Among these, 15 were HbD Punjab heterozygote showing Hb D level 31–40% and near normal RBC parameters. Four cases had HbD level 77–81.3%, with raised HbA2 levels (3.8–6%). These cases showed reduced hemoglobin, MCV, and MCH levels. They were provisionally diagnosed as double heterozygous of Hb D and beta thalassemia trait. Parental study and genetic study were done for confirmation.

Nine cases had peak in S window (RT 4.27-4.28 min), indicating presence of hemoglobin S (HbS). Eight of them had HbS level 25–40%, HbF-0.2–7.4%. Mildly raised HbA2 (3.3–3.7%) level was seen in 5 of them. There was one case with marked reduction in Hb, MCV, and MCH levels and HbA2 10% and HbS 65.4%. Parental study was advised to confirm the double heterozygous status. Sickling test was found to be positive in all these cases.

One case showed elevated P3 peak 20%, with RT 1.81 min, suggesting Hb J Meerut with reduced MCV and MCH values. Iron studies and family study were correlated.

One case showed elevated peak (RT 1.37 min), 48.8% with normal hematological parameters. It was provisionally diagnosed as Hb Hope after further confirmation by hemoglobin electrophoresis. Family study and DNA analysis were advised.

### 3.2. Discussion

India is an ethnically diverse country with marked regional variation. This diversity is reflected in the presence of different hemoglobin variants in different ethnic groups. Due to migration, there is constant mixing of peoples from different regions. Many of these abnormal variants are of little clinical significance in heterozygous state, but when combined with other variants they may give rise to severe disease. Therefore there is always a need for a screening method which can detect maximum variants. HPLC has the advantage of quantifying Hb F and Hb A2 along with detecting other variants in a single screening test.

Besides HPLC, there are other analytical procedures used for detection of thalassemia and hemoglobinopathies such as alkaline and acid electrophoresis, Hb A2 quantification by ion-exchange column chromatography, and Hb F quantification by alkali denaturation and radial immunodiffusion (9). Electrophoretic method does not separate all variants from each other, and it is recommended by screening programs such that further tests should always be carried out to confirm the presumed identity of an abnormal variant. None of the above-mentioned methods can detect multiple hemoglobin fractions in a single step procedure. HPLC has many advantages over these methods and over the past decades it has evolved as an excellent and powerful diagnostic tool for identification of most of the clinically significant Hb variants especially to beta thalassemia trait owing to its quantitative power and automation. HPLC is sensitive, specific, reproducible, and less time consuming and requires less man power. Hence, it is ideal for a routine clinical laboratory with high work load.

Our study was carried out in a tertiary care hospital in Delhi, which represented not only north Indian population but a large migrant population of eastern and north eastern parts of the country also. Apart from *β*-thalassaemia, common variants were encountered with various incidences: HbE, HbD Punjab, and HbS—being the most common along with a rare variant Hb Hope.

Thalassemia being the major concern in this study, quantitation of HbA2 and Hb F levels by HPLC was of prime importance in our laboratory where facilities for genetic studies are not available. However, parental study is also of great help in arriving at a conclusive diagnosis before referring patients for costly genetic studies.

HbA2 is constantly elevated in heterozygous beta thalassemia carriers with values ranging from 3.5 to 7% with a mean of 5% [1]. During routine reporting, we faced certain problems, regarding the cut off value of HbA2 for beta thalassemia trait. Different authors have established different cut off values for HbA2 for diagnosis of beta thalassemia trait, which ranges from 3.5 to 4%, although it has been recommended that each laboratory needs to establish their own normal ranges [4, 11]. Rangan et al. used the term borderline to HbA2 levels 3.0-4.0% and found mutations in 32% people with HbA2 3.4–3.9% [12]. Similar findings are described by Colah et al. [11]. In regions with high prevalence of beta thalassemia researchers have taken variable values as borderline, for example, 3.3–3.7% [13] and 3.1–3.9% [14].

Iron deficiency anaemia is a very common occurrence in most of the screening populations, namely, school children and pregnant women in India. There are several studies regarding the impact of iron deficiency on HbA2 level and controversy over its significance in screening of beta thalassemia trait [4, 15, 16]. Like Denic et al., we also suggest that concurrent iron deficiency anaemia should be considered in cases of borderline HbA2 with microcytic hypochromic anemia. On the other hand, we came across few cases with 3.4–3.6% HbA2 with normal MCV and MCH values. It is difficult to determine whether they are carriers of silent mutations or high normal HbA2 without genetic test. In our laboratory, range of HbA2 value with normal RBC parameter was 2.0–3.3%. Few cases with macrocytic RBC indices had values as high as 3.4%.

The variation of cut off value as well as borderline value by the same method leads to confusion resulting in underdiagnosis or overdiagnosis. In such situations, genetic counseling with DNA analysis should be recommended. But in a resource-limited country where population is huge but facilities of genetic or molecular tests are available only in a few research laboratories, we may refer only antenatal cases for genetic studies if one partner is a trait. For other cases, we can opt for parental study if possible or iron studies before referring them for costly genetic test.

On the other hand, there were few cases with symptomatic refractory microcytic hypochromic anaemia with borderline, normal, or reduced HbA2 levels. These cases should be investigated for presence of alpha thalassemia or its coinheritance with beta thalassemia gene. Alpha thalassemia is by far the commonest hemoglobinopathy in India, with highest prevalence in Punjabi population in the northern region [17]. Molecular genotyping of α-thalassemia helps to diagnose unexplained microcytosis and thus prevents unnecessary iron supplementation [18].

Hb E, the most common structural variant in our study, is one of the world's important mutations. Hb E trait, homozygous Hb E disease (Hb EE), and Hb E beta thalassemia are common in north eastern part of the country [19]. Hb E trait and Hb EE are mild disorders. Detection of this variant is very important because when combined with thalassemia or HbS, it gives rise to moderate to severe disease.

We observed that distinction between homozygous HbE disease and HbE beta thalassemia sometimes become difficult as both of these conditions show variably elevated HbE and Hb F with marked microcytic hypochromic picture. Hb D Iran also comes as a differential diagnosis. Compared to Hb E trait, Hb D Iran tends to have more area percentage at the window of Hb A2 (usually more than 40%). Parental study, if possible, may easily resolve the problem. Otherwise, genetic study should be done.

Hb D Punjab was the second most common structural variant in our study, mostly presented as asymptomatic heterozygous condition with normal hematological parameters. Hb D Punjab occurs with greatest prevalence, that is, 2% among Sikhs in Punjab, and in Gujarat, reported prevalence is 1% [20]. Hb D Punjab in the form of heterozygote Hb D trait, Hb S-D disease, and Hb D-thalassemia are commoner forms; however, homozygous form is very rare [20, 21]. Few detailed studies are available on clinical, hematological, and molecular analyses of Hb D Punjab in India [21, 22].

It has been reported that coinheritance of beta thalassemia and HbD Punjab may result in symptomatic disease and its detection is important in prenatal diagnosis. In cases, where HPLC or Hb electrophoresis shows very high HbD level and negligible HbA, one should look for raised HbA2 level and do parental study or DNA analysis for confirmation of coinheritance.

A total of nine cases of Hb S were detected of which 5 cases showed elevated Hb A2 level (3.3−3.7%) with 25–40% HbS and moderate to severe anaemia. The mean values of HbA2 have been reported to be elevated in sickle cell syndrome in previous reports [23, 24]. The reason may be HbS adducts (carbamylated and glycated) coeluting with HbA2. Parental study should be done in suspicious cases before reporting such case as sickle-beta thalassemia.

We reported 3 cases of delta-beta thalassemia trait. Delta-beta thalassemia and hereditary persistence of fetal hemoglobin (HPFH) constitute a heterogeneous group of disorders characterized by absent or reduced synthesis of adult hemoglobin (Hb A) and increased synthesis of fetal hemoglobin (Hb F). The distinction between HPFH and delta-beta thalassemia is subtle and should be confirmed by alpha-beta-globin chain synthesis ratio and DNA analysis since the distinction between these two conditions is not always possible from routine hematologic analyses. It is important to differentiate between these two conditions especially in antenatal screening because HPFH is clinically asymptomatic, but interaction of *δβ*-thalassemia with *β*-thalassemia can result in a severe disorder.

Hb J Meerut was another rare variant detected in our study. This clinically asymptomatic variant has been reported to interfere with HbA1c estimation [25] and to mask beta thalassemia trait [26].

Among the rarely encountered variants we detected one case of Hb Hope. In cation exchange HPLC method, it may be mistaken as high HbA1c, as it comes in the same position as HbA1c. Hb Hope (beta 136(H14) Gly → Asp (GGT → GAT)) is one of the unstable haemoglobin variants of the beta-globin chain, which has been demonstrated in people of various ethnic backgrounds. Few case reports of Hb hope and its association with thalassemia and Hb E have been published from southeast Asia [27, 28]. This variant is clinically silent and when associated with thalassemia may produce mild to moderate symptoms depending upon genotype.

It has been reported that one can detect HbH form of alpha thalassemia on HPLC by visual analysis of the chromatogram plot as it produces a sharp peak before the start of integration [29]. We, however, did not find any such case.

This automated HPLC system is intended for separation and determination of area percentage for HbA2 and HbF and for qualitative detection of abnormal hemoglobins. With the integration of proper algorithms involving retention time, % Hb, and peak characteristics, a clinical laboratory is capable of identifying 75% of the common variants encountered without the need for confirmatory studies such as alkaline and acid electrophoresis [9]. In the light of family study, ethnicity and clinical data, we can detect most of the frequently occurring clinically significant variants by HPLC method alone.

HPLC has some limitations, including falsely decreased HbA2 levels in patients with the HbD Punjab trait, falsely increased HbA2 levels in patients with HbS, and coelution of various Hbs, including HbE, Hb Osu Christianborg, HbG Coushatta, and Hb Lepore with HbA2 [30]. Interference from endogenous compounds or from drugs is not frequently reported in literature. Howanitz et al. reported unknown tall peaks with elution times and shapes of hemoglobin Barts on hemoglobin chromatograms that could not be confirmed by alkaline and acid gel electrophoresis mostly in patients with hemoglobin SS [31]. The authors provided evidence that the peak is not hemoglobin Barts, but rather bilirubin, and recommended exclusion of bilirubin before chromatographic results are interpreted as consistent with hemoglobin Barts. Determination of HbA2 and HbF is not interfered by endogenous substances like triglyceride and bilirubin levels up to 4600 mg/dL and 20 mg/dL, respectively [10]. In diabetic patient labile HbA1c greater than 2.5% may adversely affect HbF quantitation [10]. In our study we did not experience such interference.

## 4. Conclusion

To conclude, RBC indices, HPLC finding, and family study are sufficient to detect and manage most of the hemoglobin variants prevalent in this country. However, one has to be aware of the limitations and problems associated with the diagnostic methods to avoid false negative diagnosis in day to day practice. Genetic studies are indicated to confirm borderline cases and to detect silent carriers of beta thalassemia, alpha thalassemia, and rare and novel variants in routine practice. The present study conducted using HPLC reflects the magnitude of thalassemia and hemoglobinopathies in a small hospital based population which may be in fact the tip of an iceberg, but this type of study can definitely help to increase awareness among both health care givers and general population.

## Figures and Tables

**Figure 1:** (a) Chromatogram of beta thalassemia trait showing elevated HbA2 5.6% (RT 3.68 min) and HbF 0.4%. (b) Chromatogram showing elevated Hb F (29.1%) suggestive of HPFH.

**Figure 2:** (a) Chromatogram of HbE trait showing HbA2 24.8% (RT 3.72 min). (b) Chromatogram of E beta thalassemia showing elevated HbA2 51.4%, Hb F 30%.

**Figure 3:** (a) Chromatogram of HbE homozygous showing HbA2 77.5% (RT 3.73 min). (b) Chromatogram of Hb S trait showing Hb S 25.9% (RT 4.42 min).

**Figure 4:** (a) Chromatogram of HbD Punjab trait showing HbD 40.5% (RT 4.15 min). (b) Chromatogram of Hb D Punjab homozygous showing Hb D 87.9%.

**Figure 5:** (a) Chromatogram of showing HbA2 10.1% presumptive diagnosis of Hb Lepore. (b) Chromatogram of Hb D Iran showing HbA2 41%.

**Figure 6:** (a) Chromatogram of Hb Hope showing elevated P2 peak (48.4%). (b) Chromatogram of Hb J showing elevated P3 peak.

**Table 1:** Distribution of hemoglobin variants.

Hemoglobin variant	Number (%)
Beta thalassemia trait (BTT)	216 (74.48)
Beta thalassemia intermedia/major (BTI/M)	9 (3.10)
Hb E trait (HbAE)	28 (9.65)
Hb E disease (HbEE)	2 (0.69)
Hb E beta thalassemia (HbE-BT)	2 (0.69)
Hb D trait (HbAD)	15 (5.17)
HbD-beta thalassemia (HbD-BT)	4 (1.38)
HbS trait (HbAS)	9 (3.10)
Delta beta thalassemia (deltaBTT)	3 (1.03)
Hb J Meerut	1 (0.34)
Hb Hope	1 (0.34)

Total	290

**Table 2:** Mean values (mean ± SD) of red cell parameters and hemoglobin fractions in variants detected by HPLC.

Hb (g/dL)	RBC ×10^6^ cumm	MCV (fL)	MCH (pg)	MCHC (g/dL)	HbA (%)	HbA2 (%)	HbF (%)	Other (%)	Hb variant
10.0 ± 2.1	4.8 ± 1.02	70.7 ± 9.7	21.05 ± 3.2	29.7 ± 2.7	89.0 ± 2.5	5.2 ± 0.75	1.08 ± 0.7		BTT
4.78 ± 3.4	2.2 ± 1.3	73.2 ± 5.1	20.9 ± 2.1	28.5 ± 2.8	23.5 ± 22.6	4.06 ± 1.2	64 ± 28.6		BTM/I
10.7 ± 2.4	4.2 ± 1.05	81.8 ± 1.2	25.3 ± 3.4	31.5 ± 2.2	60.9 ± 6.6	26.6 ± 4.5	1.08 ± 1.2		HbAE
11.6 ± 1.0	5.9 ± 0.7	60.4 ± 0.7	19.8 ± 1.5	32.3 ± 2.1	3.8 ± 0.86	79.9 ± 2.5	3.92 ± 0.1		HbEE
8.5 ± 1.9	5.16 ± 1.5	63.4 ± 2.3	20.8 ± 1.3	30.3 ± 2.3	17.5 ± 9.65	61.6 ± 8.1	9.75 ± 4.7		HbE-BT
11.6 ± 2.0	4.3 ± 0.41	81.4 ± 7.3	26.2 ± 3.5	32.2 ± 2.8	52.4 ± 2.6	2.14 ± 0.5	1.02 ± 1.6	HbD36.7 ± 2	HbAD
9.65 ± 1.6	4.4 ± 0.97	67.9 ± 4.3	21.8 ± 1.8	32.1 ± 0.7	3.95 ± 2.3	4.67 ± 0.87	3.95 ± 2.3	HbD 79.7 ± 1.6	HbD-BT
9.6 ± 3.4	3.8 ± 1.4	79.6 ± 13.3	23.7 ± 5.16	30.4 ± 2.03	30.4 ± 2.03	3.25 ± 0.4	2.4 ± 2.9	HbS 29.7 ± 10.4	HbAS
11.7 ± 0.46	4.9 ± 0.49	76.3 ± 3	23.3 ± 1.5	31.4 ± 0.17	75.3 ± 0.19	2.43 ± 0.17	15.7 ± 2.6		deltaBTT
5.9	4.23	66.9	13.9	20.8	75.2	2	1.1	P3 20.0	Hb J Meerut
16.7	5.31	94.5	31.4	33.3	44.8	2.0	<1	P2 48.8	Hb Hope

**Table 3:** Genotypes of some common structural variants.

Abnormal variants	Genotype
Hb E	beta26(B8)Glu → Lys, GAG → AAG
Hb D Punjab	beta121(GH4)Glu → Gln, GAA → CAA
Hb S	beta6(A3)Glu → Val, GAG → GTG
Hb D Iran	beta22Glu → Gln, GAA → CAA
Hb Hope	beta136(H14)Gly → Asp (GGT → GAT)
Hb OArab	beta121(GH4)Glu → Lys, (GAA → AAA)
Hb C	beta6(A3)Glu → Lys, GAG → AAG
Hb J Meerut	alpha120(H3)Ala → Glu, GCG → GAG
Hb Q India	alpha64(E13)Asp → His, GAC → CAC

## References

[1] Weatherall D. J., Clegg J. B. (2001). *The Thalassemia Syndromes*.

[2] Wild B. J., Stephens A. D. (1997). The use of automated HPLC to detect and quantitate haemoglobins. *Clinical and Laboratory Haematology*.

[3] Ou C. N., Rognerud C. L. (2001). Diagnosis of hemoglobinopathies: Electrophoresis vs. HPLC. *Clinica Chimica Acta*.

[4] Rao S., Kar R., Gupta S. K., Chopra A., Saxena R. (2010). Spectrum of haemoglobinopathies diagnosed by cation exchange-HPLC & modulating effects of nutritional deficiency anaemias from north India. *Indian Journal of Medical Research*.

[5] Mohanty D., Colah R. B., Gorakshakar A. C. (2013). Prevalence of *β*-thalassemia and other haemoglobinopathies in six cities in India: a multicentre study. *Journal of Community Genetics*.

[6] Sachdev R., Dam A. R., Tyagi G. (2010). Detection of Hb variants and hemoglobinopathies in Indian population using HPLC: report of 2600 cases. *Indian Journal of Pathology and Microbiology*.

[7] Ou C. N., Buffone G. J., Reimer G. L., Alpert A. J. (1983). High-performance liquid chromatography of human hemoglobins on a new cation exchanger. *Journal of Chromatography*.

[8] Kutlar A., Kutlar F., Wilson J. B. (1984). Quantitative of hemoglobin components by high-performance cation-exchange liquid chromatography: its use in diagnosis and in the assessment of cellular distribution of hemoglobin variants. *American Journal of Hematology*.

[9] Joutovsky A., Hadzi-Nesic J., Nardi M. A. (2004). HPLC retention time as a diagnostic tool for hemoglobin variants and hemoglobinopathies: a study of 60000 samples in a clinical diagnostic laboratory. *Clinical Chemistry*.

[11] Colah R. B., Surve R., Sawant P. (2007). HPLC studies in hemoglobinopathies. *Indian Journal of Pediatrics*.

[12] Rangan A., Sharma P., Dadu T., Saxena R., Verma I. C., Bhargava M. (2011). B-Thalassemia mutations in subjects with borderline HbA 2 values: a pilot study in North India. *Clinical Chemistry and Laboratory Medicine*.

[13] Mosca A., Paleari R., Galanello R. Occurrence of HbA2 borderlinephenotypes in areas with high prevalence of thalassemia.

[14] Giambona A., Passarello C., Vinciguerra M. (2008). Significance of borderline hemoglobin A2 values in an Italian population with a high prevalence of *β*-thalassemia. *Haematologica*.

[15] Passarello C., Giambona A., Cannata M., Vinciguerra M., Renda D., Maggio A. (2012). Iron deficiency does not compromise the diagnosis of high HbA2 *β* thalassemia trait. *Haematologica*.

[16] Denic S., Agarwal M. M., Al Dabbagh B. (2013). Hemoglobin A_2_ lowered by iron deficiency and α-thalassemia: should screening recommendation for *β*-thalassemia change?. *ISRN Hematology*.

[17] Nadkarni A., Phanasgaonkar S., Colah R., Mohanty D., Ghosh K. (2008). Prevalence and molecular characterization of alpha-thalassemia syndromes among Indians. *Genetic Testing*.

[18] Sankar V. H., Arya V., Tewari D., Gupta U. R., Pradhan M., Agarwal S. (2006). Genotyping of alpha-thalassemia in microcytic hypochromic anemia patients from North India. *Journal of Applied Genetics*.

[19] Mohanty D., Colah R. B., Gorakshakar A. C. (2013). Prevalence of *β*-thalassemia and other haemoglobinopathies in six cities in India: a multicentre study. *Journal of Community Genetics*.

[20] Lukens J. N., Lee G. R., Foerster J., Lukens J., Paraskevas F., Greer J. P., Rodgers G. M. (1998). The abnormal hemoglobins: general principles. *Wintrobe's Clinical Hematology*.

[21] Pandey S., Mishra R. M., Pandey S., Shah V., Saxena R. (2012). Molecular characterization of hemoglobin D Punjab traits and clinical-hematological profile of the patients. *Sao Paulo Medical Journal*.

[22] Srinivas U., Pati H. P., Saxena R. (2010). Hemoglobin D-Punjab syndromes in India: a single center experience on cation-exchange high performance liquid chromatography. *Hematology*.

[23] Shokrani M., Terrell F., Turner E. A., del Pilar Aguinaga M. (2000). Chromatographic measurements of hemoglobin A2 in blood samples that contain sickle hemoglobin. *Annals of Clinical & Laboratory Science*.

[24] Suh D. D., Krauss J. S., Bures K. (1996). Influence of hemoglobin S adducts on hemoglobin A_2_ quantification by HPLC. *Clinical Chemistry*.

[25] Sharma A., Marwah S., Buxi G., Yadav R. B. (2012). Falsely low HbA1c value due to a rare hemoglobin variant (Hemoglobin J-Meerut) - A family study. *Indian Journal of Pathology and Microbiology*.

[26] Giordano P. C., Maatman R. G., Niessen R. W., van Delft P., Harteveld C. L. (2006). Beta thalassemia IVS-I-5(G→C) heterozygosity masked by the presence of HbJ-Meerut in a Dutch-Indian patient. *Haematologica*.

[27] Chunpanich S., Fucharoen S., Sachaisuriya K., Fucharoen G., Kam-Itsara K. (2004). Molecular and hematological characterization of hemoglobin hope/hemoglobin E and hemoglobin hope/α-Thalassemia 2 in Thai patients. *Laboratory Hematology*.

[28] Sura T., Busabaratana M., Youngcharoen S., Wisedpanichkij R., Viprakasit V., Trachoo O. (2007). Haemoglobin Hope in a Northern Thai family: first identification of homozygous haemoglobin Hope associated with haemoglobin H disease. *European Journal of Haematology*.

[29] Wadhwa R., Singh T. (2011). Role of HPLC in the detection of HbH disease. *Indian Journal of Pathology and Microbiology*.

[30] Higgns T. N., Khajuria A., Mack M. (2009). Quantification of HbA2 in patients with and without *β*-thalassemia and in the presence of HbS, HbC, HbE, and HbD Punjab hemoglobin variants: comparison of two systems. *The American Journal of Clinical Pathology*.

[31] Howanitz P. J., Kozarski T. B., Howanitz J. H., Chauhan Y. S. (2006). Spurious hemoglobin Barts caused by bilirubin: a common interference mimicking an uncommon hemoglobinopathy. *The American Journal of Clinical Pathology*.

